# Loss of pigment epithelium-derived factor: a novel mechanism for the development of endocrine resistance in breast cancer

This article has been retracted.

**DOI:** 10.1186/bcr3356

**Published:** 2012-11-14

**Authors:** Rifat Jan, Min Huang, Joan Lewis-Wambi

**Affiliations:** 1 Cancer Biology Program, The Research Institute of Fox Chase Cancer Center, 333 Cottman Avenue, Philadelphia, PA 19111, USA; 2 Department of Pathology, The Research Institute of Fox Chase Cancer Center, 333 Cottman Avenue, Philadelphia, PA 19111, USA

## Abstract

**Introduction:**

Despite the benefits of endocrine therapies such as tamoxifen and aromatase inhibitors in treating estrogen receptor (ER) alpha-positive breast cancer, many tumors eventually become resistant. The molecular mechanisms governing resistance remain largely unknown. Pigment epithelium-derived factor (PEDF) is a multifunctional secreted glycoprotein that displays broad anti-tumor activity based on dual targeting of the tumor microenvironment (anti-angiogenic action) and the tumor cells (direct anti-tumor action). Recent studies indicate that PEDF expression is significantly reduced in several tumor types, including breast cancer, and that its reduction is associated with disease progression and poor patient outcome. In the current study, we investigated the role of PEDF in the development of endocrine resistance in breast cancer.

**Methods:**

PEDF mRNA and protein levels were measured in several endocrine-resistant breast cancer cell lines including MCF-7:5C, MCF-7:2A, and BT474 and in endocrine-sensitive cell lines MCF-7, T47D, and ZR-75-1 using real-time PCR and western blot analyses. Tissue microarray analysis and immunohistochemistry were used to assess the PEDF protein level in tamoxifen-resistant breast tumors versus primary tumors. Lentiviruses were used to stably express PEDF in endocrine-resistant breast cancer cell lines to determine their sensitivity to tamoxifen following PEDF re-expression.

**Results:**

We found that PEDF mRNA and protein levels were dramatically reduced in endocrine-resistant MCF-7:5C, MCF-7:2A, and BT474 breast cancer cells compared with endocrine-sensitive MCF-7, T47D, and ZR-75-1 cells, and that loss of PEDF was associated with enhanced expression of p^Ser167^ERα and the receptor tyrosine kinase rearranged during transfection (RET). Importantly, we found that silencing endogenous PEDF in tamoxifen-sensitive MCF-7 and T47D breast cancer cells conferred tamoxifen resistance whereas re-expression of PEDF in endocrine-resistant MCF-7:5C and MCF-7:2A cells restored their sensitivity to tamoxifen *in vitro *and *in vivo *through suppression of RET. Lastly, tissue microarray studies revealed that PEDF protein was reduced in ~52.4% of recurrence tumors (31 out of 59 samples) and loss of PEDF was associated with disease progression and poor patient outcome.

**Conclusion:**

Overall, these findings suggest that PEDF silencing might be a novel mechanism for the development of endocrine resistance in breast cancer and that PEDF expression might be a predictive marker of endocrine sensitivity.

## Introduction

The female hormone estrogen has long been recognized as being important for stimulating the growth of a large proportion of breast cancers. Estrogen action is mediated by two receptors; estrogen receptor (ER) alpha and ER beta. Approximately 70% of breast cancers express ERα [1,2], and its presence in breast tumors is routinely used to predict a response to endocrine therapy such as tamoxifen - an anti-estrogen that blocks estrogen-stimulated breast cancer cell growth - or aromatase inhibitors (AIs) - agents that suppress estrogen synthesis in the body. These agents are highly effective and are less toxic compared with chemotherapy, and are often offered to ER-positive breast cancer patients to sustain a better quality of life [3,4]. Despite the clinical benefits of tamoxifen and AIs, however, a large number of breast cancer patients develop drug resistance. It is estimated that ~40% of patients with early ER-positive breast cancer relapse within 15 years after adjuvant therapy with tamoxifen and 15% of patients treated with an AI relapse within 9 years [5-7]. These resistant tumors are usually more aggressive and are more likely to metastasize, which is often the leading cause of breast cancer-related death. There is strong evidence that endocrine resistance is associated with cross-talk between upstream kinases and ERα, resulting in estrogen-independent activation of the ERα; however, the exact mechanism by which breast cancer cells develop resistance to endocrine therapy is still not fully understood.

Pigment epithelium-derived factor (PEDF) is a 50 kDa glycoprotein that belongs to the non-inhibitory serine protease inhibitor superfamily but it does not inhibit proteases [8,9]. PEDF was first discovered as a factor secreted by retinal pigment epithelial cells [10], but was later found to be expressed in several tissues including the brain, spinal cord, eye, plasma, bone, prostate, pancreas, heart and lung [11]. PEDF is present in human blood at a concentration of approximately 100 nM (5 μg/ml) or twice the level required to inhibit aberrant blood-vessel growth in the eye [10]. PEDF possesses potent anti-angiogenic activity, far greater than any other known anti-angiogenic factor [12], and it has anti-tumor properties including the ability to promote tumor differentiation and initiate apoptosis [13-16]. In endothelial cells, PEDF has been shown to induce apoptosis by activating the Fas/Fas-L caspase-8 apoptotic pathway [17,18] and there is evidence that the p38 mitogen-activated protein kinase (MAPK) pathway is involved in the anti-angiogenic activity of PEDF [19]. More recently, a number of studies have reported that PEDF expression is significantly reduced in several tumor types, including prostate adenocarcinoma [20], pancreatic adenocarcinoma [21], glioblastoma [22], ovarian carcinoma [23], and breast cancer [24]. With regards to breast cancer, PEDF expression has been shown to be markedly reduced in breast tumors compared with normal tissue and this reduction is associated with disease progression and poor patient outcome [24,25]. At present, however, it is not known whether PEDF plays a role in the development of endocrine resistance.

In this study, we examined the role of PEDF in the development of endocrine resistance using several breast cancer cell lines. Specifically, we evaluated PEDF expression in endocrine-resistant MCF-7:5C, MCF-7:2A, and BT474 breast cancer cells versus endocrine-sensitive MCF-7, T47D, and ZR-75-1 cells and found that PEDF mRNA and protein levels were dramatically reduced in the endocrine-resistant breast cancer cell lines compared with the endocrine-sensitive cell lines. In addition, tissue microarray studies revealed that PEDF protein was significantly reduced in tamoxifen-resistant/recurrence tumors compared with primary tumors. We also found that re-expression of PEDF in endocrine-resistant MCF-7:5C and BT474 cells restored their sensitivity to tamoxifen, whereas siRNA knockdown of PEDF in MCF-7 and T47D cells markedly reduced their sensitivity to tamoxifen. Notably, re-expression of PEDF in endocrine-resistant MCF-7:5C cells resulted in a significant reduction in the level of p-ERα, p-AKT, and rearranged during transfection (RET) proteins, which were constitutively overexpressed in these cells. Lastly, we found that recombinant PEDF (rPEDF) dramatically reduced the tumor growth of MCF-7:5C xenographs in athymic mice and that re-expression of PEDF in MCF-7:5C cells partially restored tamoxifen sensitivity *in vivo*. Taken together, these findings suggest that PEDF silencing might be a novel mechanism for the development of endocrine resistance in breast cancer.

## Materials and methods

### Cell lines and culture conditions

The MCF-7 cells used in this study [26] were cloned from ERα-positive human MCF-7 breast cancer cells originally obtained from the American Type Culture Collection (Manassas, VA, USA). MCF-7 cells were maintained in full serum medium composed of RPMI-1640 medium, 10% fetal bovine serum, 2 mM glutamine, penicillin at 100 U/ml, streptomycin at 100 μg/ml, 1× nonessential amino acids (Invitrogen, Grand Island, NY, USA), and bovine insulin at 6 ng/ml (Sigma-Aldrich, St Louis, MO, USA). ER-positive MCF-7:5C [27,28] and MCF-7:2A [29,30] breast cancer cells were cloned from MCF-7 cells following long-term (> 12 months) culture in estrogen-free medium composed of phenol red-free RPMI, 10% fetal bovine serum treated three times with dextran-coated charcoal, 2 mM glutamine, bovine insulin at 6 ng/ml, penicillin at 100 U/ml, streptomycin at 100 μg/ml, and 1× nonessential amino acids. MCF-7:5C cells are resistant to AIs (that is, hormone independent) and tamoxifen, but these cells undergo apoptosis in the presence of physiologic concentrations of 17β-estradiol (E2), as previously reported [28]. MCF-7:2A cells are also resistant to AIs but only partially sensitive to tamoxifen, and these cells undergo apoptosis in the presence of E2 [29,31].

The human breast cancer cell line T47D:A18, referred to as T47D in this study, is a hormone-responsive clone of wild-type T47D that has been described previously [32]. These cells were maintained in phenol red-containing RPMI medium supplemented with 10% fetal bovine serum (FBS), bovine insulin (6 ng/ml), and antibiotics. ER-positive ZR-75-1 and BT474 breast cancer cells were obtained from the American Type Culture Collection and were maintained in phenol red-containing RPMI medium supplemented with 10% FBS, bovine insulin (6 ng/ml), and antibiotics. The BT474 cell line was isolated by Lasfargues and Coutinho from a solid, invasive ductal carcinoma of the breast [33]. ER-negative MDA-MB-231 breast cancer cells were obtained from the American Type Culture Collection and were cultured in DMEM medium supplemented with 10% FBS and antibiotics.

MCF-7:5C cells stably expressing PEDF (5C-PEDF) were grown in phenol red-free RPMI 1640 medium supplemented with 10% phenol red-free RPMI, 10% fetal bovine serum treated three times with dextran-coated charcoal and 4 μg/ml blasticidin (InvivoGen, San Diego, CA, USA), and BT474 cells stably expressing PEDF (BT474-PEDF) were grown in RPMI medium supplemented with 10% FBS and 4 μg/ml blasticidin (InvivoGen, San Diego, CA, USA).

### Cell proliferation assay

This procedure has been described previously [28,29,34]. Briefly, MCF-7 and T47D cells were grown in fully estrogenized medium. Cells were seeded in 24-well plates (30,000/well) and after overnight incubation were transfected with either control (nontarget) or PEDF siRNA. Transfected cells were treated with 10^-6 ^M 4-hydroxytamoxifen (4OHT) after 48 hours, and then cells were harvested after 72 hours and total DNA was determined using a Fluorescent DNA Quantitation kit (Bio-Rad Laboratories, Hercules, CA, USA), as previously described [28]. Cell proliferation was also determined by cell counting using the trypan blue exclusion assay. MCF-7 and T47D cells were seeded in six-well plates (1 × 10^5^/well) and then treated with 10^-6 ^M 4OHT for 72 hours. The 4OHT used in the cell proliferation studies was purchased from Sigma-Aldrich.

We also performed proliferation studies using MCF-7:5C, BT474, 5C-PEDF, and BT474-PEDF cells. MCF-7:5C and 5C-PEDF cells were grown in non-estrogenized media, and BT474 and BT474-PEDF cells were grown in fully estrogenized media. For the DNA proliferation assay, cells were seeded at a density of 30,000/well in 24-well plates and after overnight incubation were treated with 10^-12 ^M to 10^-6 ^M 4OHT for 7 days with retreatment on alternate days. Cells were then harvested and total DNA quantitated using a Fluorescent DNA kit as described previously [28]. For cell counting, cells were seeded at 75,000/well in six-well plates and after overnight incubation were treated with 10^-6 ^M 4OHT for 72 hours. Cells were then harvested and counted using trypan blue exclusion.

### Western blot analysis

Immunoblotting was performed using 30 μg protein per well as described previously [28,35]. Membranes were probed with primary antibodies against PEDF (Chemicon Inc., Temecula, CA., USA), against ERα and phospho-Ser167-ERα (Santa Cruz Biotechnology, Inc., Santa Cruz, CA, USA), against RET, p-RET (Y1062), mammalian target of rapamycin (mTOR), p-mTOR and AKT, and against pAKT, MAPK, pMAPK and p70S6K (Cell Signaling Technology Inc., Danvers, MA, USA), and against β-actin (Sigma Chemical Co., St Louis, MO, USA). The appropriate secondary antibody conjugated to horseradish peroxidase (Santa Cruz Biotechnology) was used to visualize the stained bands with an enhanced chemiluminescence visualization kit (Amersham, Arlington Heights, IL, USA). Bands were quantitated by densitometry using the Molecular Dynamics Software ImageQuant (GE Healthcare Life Sciences, Piscataway, NJ, USA) and densitometric values were corrected for loading control.

### Knockdown of PEDF and RET with small interference RNA

For the iRNA silencing experiments, PEDF, RET, and nontarget control siRNAs were purchased from Dharmacon Inc (Pittsburg, PA, USA). For transfection, 100 nM siRNAs were combined with siRNA transfection reagent according to the manufacturer's instructions. Cells were seeded in 24-well plates at a density of 0.5 × 10^5 ^cells/well in antibiotics-free medium 12 hours before the transfection. One and a half microliters of the siRNA (20 μM) were mixed with 1 μl transfection reagent in 50 μl serum-free RPMI-1640 medium and were incubated at room temperature for 25 minutes to form a complex. After washing cells with PBS, the 50 μl transfection mixtures were added to each well with 450 μl RPMI-1640 medium containing 10% FBS at a final concentration of 100 nM siRNA. Twenty-four hours after the transfection, the medium was replaced with fresh 500 μl RPMI-1640 medium containing 10% FBS. Transfected cells were then harvested for western blotting and RT-PCR or subsequently treated with 10^-9 ^M to 10^-6 ^M 4OHT for 3 days to determine cell growth.

### RNA isolation and RT-PCR analysis

Total RNA was isolated from cultured cells using the TRIzol reagent (Invitrogen) according to the manufacturer's procedure. First-strand cDNA synthesis was performed from 2.5 μg total RNA using Super-Script Reverse Transcriptase (Invitrogen). cDNA was amplified in a 15-μl PCR mixture containing 1 mm dNTPs, 1× PCR buffer, 2.5 mm MgCl_2_, and 1 U DNA *Taq *polymerase (Promega, Madison, WI, USA) with 25 pmol of primers specific for human *PEDF *(sense, 5'-CATTCACCGGGCTCTCTAC-3'; antisense, 5'-GGCAGCTGGGCAATCTTGCA-3') and human *RET *(sense, 5'-GGATTTCGGCTTGTCCCGAG-3'; antisense, 5'-CCATGTGGAAGG GAGGGCTC-3'). The conditions in the logarithmic phase of PCR amplification were as follows: 5 minutes initial denaturation at 94°C, 1 minute denaturation at 94°C, 35 seconds annealing at 67°C, and 1.5 minute extension at 72°C for 30 cycles. The number of amplification cycles during which PCR product formation was limited by the template concentration was determined in pilot experiments. *PUM1 *was used as the internal control (sense, 5'-TCACCGAGGCCCCTCTGAACCCTA-3'; antisense, 5'-GGCAGTAATC TCCTTCTGCATCCT-3').

The reproducibility of the quantitative measurements was evaluated by three independent cDNA syntheses and PCR amplification from each preparation of RNA. Densitometric analysis was performed using Scion Image software (Scion Corp., Frederick, MD, USA), and the relative *PEDF *or *RET *mRNA expression levels were determined as the ratio of the signal intensity of PEDF to that of *PUM1*.

### Estrogen response element luciferase assay

To determine ERα transcriptional activity, cells were transfected with an estrogen response element (ERE)-regulated (pERE(5×)TA-ffLuc plus pTA-srLuc) dual-luciferase reporter gene set. pERE(5×)-ffLuc contained five copies of a consensus ERE and a TATA-box driving firefly luciferase; pTATA-srLuc contained a TATA-box element driving renilla luciferase. Cells were grown in the estrogen-free medium containing no exogenous compounds for 2 days before transfection. All transfection experiments were carried-out using LT1 (Mirus Bio LLC, Madison, WI, USA) at a 1:3 ratio of micrograms of plasmid to micoliters of LT1. In the ERE reporter gene experiment, the cells were treated as indicated 24 hours following the transfection. Forty-eight hours following the ERE transfection, the cells were harvested and processed for dual-luciferase reporter activity (Promega, Madison, WI, USA), in which the firefly luciferase activity was normalized by renilla luciferase activity.

### Breast cancer tissue microarray and immunohistochemistry

Paraffin-embedded de-identified human breast cancer tissue samples were collected from the Tumor Bank facility at the Fox Chase Cancer Center and the protocols were reviewed and approved by the Institutional Review Board at our institution. The archived tumor samples were obtained from patients who were initially treated with tamoxifen and either responded (*n *= 150) or responded but then developed recurrence disease (*n *= 59) with an average time to disease progression of 93 months. Patients provided written informed consent for the use of their tumor samples.

Tissue microarray slides were constructed from 59 matching primary and recurrence tumors using duplicate cores of 0.6 mm per tumor sample. Tissue microarray slides were also created using endocrine-responsive tumors. For PEDF and ERα immunohistochemistry, sections were incubated at room temperature for 20 minutes with anti-PEDF or anti-ERα antibody (Chemicon Inc.) applied at 1:100 dilution in antibody diluent (Dako USA, Carpinteria, CA, USA). A secondary anti-mouse antibody polymer conjugated with horseradish peroxidase (Dako USA) was applied for 30 minutes and 3,3'-diaminobenzidine was used to produce visible, localized staining viewable with light microscopy. Sections without primary antibody served as negative controls. Normal breast tissue from archival specimens was used as positive controls for PEDF and ERα expression. A semi-automated quantitative image analysis system (ACIS II; ChromaVision Medical Systems, Inc., San Juan Capistrano, CA, USA) was used to quantitate the staining of the tissue microarray slides. For immunohistochemical analysis, the brown stain intensity of the chromogen was compared with the blue counterstain used as background. Staining for PEDF was quantified as an intensity score (scale 0 to 255) and staining for ERα was graded as follows: 0, negative (no cells stained); 1, weakly positive (< 10% of cells stained); 2, moderately positive (10 to 50% of cells stained); or 3, strongly positive (> 50% cells stained).

### TUNEL staining for apoptosis

Apoptosis was determined by the terminal deoxynucleotidyl transferase-mediated dUTP nick end-labeling (TUNEL) assay using an *in situ *cell death detection kit (POD; Roche Molecular Biochemicals, Branchburg, NJ, USA), according to the manufacturer's instructions. Briefly, fixed cells were washed, permeabilized, and then incubated with 50 μl terminal deoxynucleotidyl transferase end-labeling cocktail for 60 minutes at 37°C in a humidified atmosphere in the dark. For signal conversion, slides were incubated with 50 μl converter-POD (anti-fluorescein antibody conjugated with horseradish peroxidase) for 30 minutes at 37°C, rinsed with PBS, and then incubated with 50 μl of 3,3'-diaminobenzidine substrate solution for 10 minutes at 25°C. The slides were then rinsed with PBS, mounted under glass coverslips, and analyzed under a light microscope (Inverted Nikon TE300; Melville, NY, USA).

### Lentiviral vector design, production, and transduction

For PEDF overexpression, we generated a lentiviral construct encoding the full-length human PEDF cDNA inserted between *Xba*I and *Bam*HI sites of the prrl.CMV.EGFP.wpre.SIN lentiviral vector. Briefly, PEDF cDNA was amplified by PCR from pCEP4-PEDF plasmid (a gift from Dr Bouck, Northwestern University, Chicago, IL, USA); *Xba*I and *Xba*I + *Eco*RV sites were added to the 5' and 3' ends, respectively, using primers 5'-CTAGTCTAGAGGCCCCAGGATGCAGGC CCTG-3' and 5'-GGCCTCTAGATATCTTAGGGGCCCCTGGGGTCCAG-3'. This fragment was then subcloned into TA cloning vector (Invitrogen, San Diego, CA, USA), digested with *Eco*RV and *Xba*I and re-cloned in the prrl.CMV.EGFP.wpre.SIN plasmid digested with *Xba*I and *Bam*HI. To produce lentiviral stock, 293FT cells (Invitrogen) were plated in 10-cm tissue culture plates. When the cells were 90 to 95% confluent, the complete culture medium was removed and the cells were exposed to 5 ml medium (Opti-MEM I; Invitrogen) with complexes (DNA-Lipofectamine 2000; Invitrogen) containing 9 μg packaging mix (ViralPower; Invitrogen), 3 μg expression plasmid DNA (prrl.CMV.EGFP.wpre.SIN/PEDF), or control plasmid DNA (prrl.CMV.EGFP.wpre.SIN/LacZ) with lipofectamine (Lipofectamine 2000; Invitrogen). Hexadimethrine bromide (Polybrene; Sigma-Aldrich) was added at the final concentration of 10 μg/ml. After incubation for 24 hours, the infection medium was replaced with complete culture medium. Lentivirus-containing supernatants were harvested 72 hours after transfection. The supernatants were centrifuged to remove pellet debris and stored at -80°C.

For lentiviral vector transduction, MCF-7:5C and BT474 cells were plated in six-well plates. When the cells reached 30 to 50% confluence, media were changed to either phenol red-free RPMI medium with 10% charcoal-stripped FBS without antibiotic (MCF-7:5C cells) or complete growth medium without antibiotic (BT474 cells) with the lentiviral stock, and 10 μg/ml hexadimethrine bromide (Polybrene; Sigma-Aldrich) was added to improve lentiviral vector transduction. Lentiviral vector expressing lacZ served as a positive control. After overnight incubation at 37°C in 5% CO_2_, the media-containing virus was removed and replaced with 2 ml complete culture media. After incubation overnight at 37°C in 5% CO_2_, media were changed to phenol red-free RPMI medium with 10% charcoal-stripped FBS without antibiotic or respective media with 4 μg/ml blasticidin (InvivoGen). Transduced cell clones were then selected with antibiotic for 2 weeks. PEDF expression was verified by quantitative real-time RT-PCR and western blot analysis in MCF-7:5C and BT474 cells.

### Animal studies

The mammary fat pads of 6-week-old to 8-week-old ovariectomized outbred athymic mice (Taconic, Upstate, NY, USA) were bilaterally inoculated with 5 × 10^6 ^MCF-7:5C cells suspended in 0.1 ml sterile PBS solution as described previously [28]. When tumors reached a mean cross-sectional area of 0.1 cm^2^, the mice were randomized into groups of 10 and were treated with sterile PBS (100 μl) or 4 mg/kg rPEDF that was administered by intraperitoneal injection for a total of 30 days. Mice were injected every 2 days and tumors were measured every 5 days with vernier calipers. The mean cross-sectional tumor area was calculated by multiplying the length (*l*) by the width (*w*) by π and dividing the product by four (that is, *lw*π/4). The mean cross-sectional tumor area was plotted against time in days to monitor tumor growth. The mice were sacrificed by CO_2 _inhalation and cervical dislocation; tumors were excised and immediately fixed in 10% buffered formalin for immunohistochemistry or snap-frozen in liquid nitrogen. Frozen tumor specimens were stored at -80°C for further analysis.

In another experiment, a total of 96 ovariectomized outbred athymic mice, 6 to 8 weeks old, were bilaterally inoculated with 5 × 10^6 ^MCF-7, BT474, or MCF-7:5C breast cancer cells suspended in 0.1 ml sterile PBS. Mice injected with MCF-7 (*n *= 32) or BT474 cells (*n *= 32) were simultaneously treated with E2 to stimulate tumor growth. E2 was administered via 0.3 cm long silastic capsules (Innovative Research, Sarasota, FL, USA) that were implanted subcutaneously between the scapules. The capsules remained in place for the duration of the study (3 to 6 weeks). Mice injected with MCF-7:5C cells (*n *= 32), however, did not require treatment with E2 because these cells are estrogen independent and are capable of forming tumors in the absence of E2, as reported previously [28]. When the mean tumor cross-sectional area reached approximately 0.3 cm^2 ^for MCF-7 and BT474-injected mice and 0.2 cm^2 ^for MCF-7:5C-injected mice, groups of eight mice were randomly assigned to the following treatments: PBS alone (control), rPEDF, tamoxifen, or tamoxifen plus rPEDF. Tamoxifen was administered orally by gavage at 1.5 mg/day per mouse for 5 days/week for 21 days and rPEDF was administered by intraperitoneal injection at 4 mg/kg every 2 days for 21 days. Tumors were measured weekly with vernier calipers. The mean cross-sectional tumor area was calculated by multiplying the length (*l*) by the width (*w*) and by π and dividing by 4 (that is, *lw*π/4).

All animal experiments were carried out according to the guidelines of the American Association for Laboratory Animal Science as an approved protocol by the Institutional Animal Care and Use Committee at the Institute for Cancer Research-Fox Chase Cancer Center.

### Microvessel density assay

Frozen tissues were cut into 10-μm sections, fixed in acetone at 4°C for 5 minutes, and blocked for endogenous peroxidase. Sections were treated with normal serum for 10 minutes. Tumor sections were incubated with the rat monoclonal antibody against mouse CD34 (BD Pharmingen, San Diego, CA, USA) at 1:100 dilutions at 4°C. After rinsing with PBS, sections were incubated with biotinylated rabbit antigoat immunoglobulins (Dako, Glostrup, Denmark) at 1:1,000 dilutions for 30 minutes at room temperature followed by incubation with horseradish peroxidase-labeled streptavidin-biotin complex for 30 minutes. The peroxidase reaction was visualized using diaminobenzidine. The tumor microvessel density was quantified as tumor vasculature. In negative-control staining, the primary antibodies were omitted.

### Statistical analysis

All *in vitro *experiments were repeated at least twice in either duplicate or triplicate with different cell preparations to ensure consistency of the findings. One-factor analysis of variance was used to demonstrate that there were significant differences between conditions when there were more than two conditions, and paired analyses were performed using either Student's *t *test or the Mann-Whitney test (GraphPad Software, San Diego, CA, USA) in order to identify the conditions that were significantly different. For *in vivo *studies, tumor growth curves were analyzed longitudinally using a two-factor analysis of variance comparing tumor cross-sectional areas within treatments in a time-dependent manner. Tumor growth curves represent the mean ± standard error of tumor cross-sectional areas. *P *< 0.05 was considered statistically significant.

## Results

### PEDF expression is dramatically reduced in endocrine-resistant breast cancer cells

To determine whether there is an association between PEDF expression and endocrine resistance, we first examined PEDF expression in a panel of breast cancer cell lines using western blot and real-time PCR analyses. We found that PEDF protein (Figure 1a) and mRNA (Figure 1b) levels were dramatically reduced in endocrine-resistant MCF-7:5C, MCF-7:2A, and BT474 breast cancer cells compared with endocrine-sensitive MCF-7, T47D, and ZR-75-1 cells with no PEDF observed in ER-negative MDA-MB-231 cells. A similar trend was observed when the media conditioned by these cells were tested for PEDF expression. As shown in Figure 1c, endocrine-sensitive T47D, ZR-75-1 and, to a lesser extent, MCF-7 cells secreted the most PEDF, whereas endocrine-resistant MCF-7:5C, MCF-7:2A, and BT474 cells secreted markedly less to no detectable level of PEDF. Interestingly, we found that tamoxifen-resistant BT474 cells expressed a level of PEDF almost comparable with that of MCF-7 cells whereas AI-resistant MCF-7:5C and MCF-7:2A cells expressed very little to no PEDF. We should note that there are differences between BT474 cells and long-term estrogen-deprived MCF-7:5C and MCF-7:2A cells. Specifically, BT474 cells overexpress HER2 and the ER coactivator AIB1, which contribute to tamoxifen resistance in these cells [36], whereas MCF-7:5C and MCF-7:2A cells express low levels of HER2 and AIB1 but high levels of phospho-Akt and ERα, which are thought to contribute to the AI-resistant and tamoxifen-resistant phenotype of these cells. Tamoxifen resistance has been studied by several groups [37,38] and is believed to be due primarily to crosstalk between ER and HER2. This crosstalk leads to enhanced cell survival pathways via phosphoinositide 3-kinase (PI3K)/AKT activation in addition to activation of various MAPKs that mediate transcriptional effects resulting in cell proliferation. In contrast, studies using long-term estrogen-deprived breast cancer cells have shown that AI resistance is controlled by several signaling pathways including the P13K/AKT pathway, the insulin-like growth factor receptor (IGF-1R) pathway, and the HER2 pathway [39-41]. In addition, we have previously shown that AI-resistant MCF-7:5C and MCF-7:2A cells undergo apoptosis in the presence of physiological concentrations of E2 [28,29,42]. The differences in PEDF expression between BT474, MCF-7:5C, and MCF-7:2A cells might possibly be influenced by the different signaling pathways that control the resistant phenotype of these cells.

**Figure 1:** **Pigment epithelium-derived factor expression in human breast cancer cell lines**. **(a) **Pigment epithelium-derived factor (PEDF) and estrogen receptor alpha (ERα) protein levels were detected by western blot analysis in several human breast cancer cell lines, including hormone-dependent T47D, MCF-7, and ZR-75-1 cells, tamoxifen-resistant BT474 cells, tamoxifen-resistant and aromatase inhibitor-resistant MCF-7:5C and MCF-7:2A cells, and ER-negative MDA-MB-231 cells. **(b) ***PEDF *mRNA expression level in the different breast cancer cell lines was determined by quantitative real-time PCR analysis with *PUM1 *used as a normalization control. **(c) **Conditioned media were analyzed by western blot for the presence of PEDF protein in the indicated breast cancer cell lines. Staining of proteins by Coomassie blue included as a loading control. **(d) **Hormonal regulation of PEDF and ERα protein in MCF-7 and T47D breast cancer cells. Cells were incubated in phenol red-free RPMI media supplemented with 10% charcoal-stripped FBS for 72 hours and, subsequently, were treated with vehicle, 1 nM 17β-estradiol (E2), or 1 nM E2 + 1 μM 4-hydroxytamoxifen (4OHT) for 24 hours, and the PEDF and ERα protein level was determined by western blot analysis. β-actin was used as a normalization control. All experiments were performed in triplicate independently.

The ERα protein level was also examined in the different cell lines to assess whether there was a correlation between ERα status and PEDF expression. Figure 1a showed that ERα protein was expressed in all of the cell lines except for MDA-MB-231 cells, which are ERα-negative; however, ERα was significantly elevated in endocrine-resistant MCF-7:5C, MCF-7:2A, and BT474 cells compared with endocrine-sensitive MCF-7, T47D, and ZR-75-1 cells. In addition, we found that E2 treatment markedly reduced the PEDF protein level in MCF-7 and T47D cells whereas 4OHT, the active metabolite of tamoxifen, significantly increased the PEDF protein level in both cell lines (Figure 1d). A similar trend was observed for ERα regulation by E2 and 4OHT in MCF-7 and T47D cells (Figure 1d). Overall, these data show that PEDF expression is significantly reduced in endocrine-resistant breast cancer cells compared with endocrine-sensitive cells and that its expression is differentially regulated by estrogen and anti-estrogen in hormone-dependent breast cancer cells. No significant correlation, however, was observed between PEDF expression and total ERα status.

### PEDF expression is dramatically reduced in endocrine-resistant breast tumors

Since PEDF expression was dramatically reduced in endocrine-resistant breast cancer cells, we next determined whether there was a clinical correlation between PEDF expression and the development of endocrine resistance in breast tumors. PEDF expression was examined in primary versus recurrence tumors. A total of 209 breast cancer patients were initially treated with tamoxifen and responded; however, 59 patients developed recurrence disease with an average time to disease progression of 93 months. Immunohistochemical staining was performed on tissue microarrays constructed using recurrence breast tumor tissues (*n *= 59) versus matched primary breast tumor tissues (*n *= 59). Figure 2a shows that PEDF protein was dramatically reduced in the recurrence breast cancer tissue (right panel) compared with the primary breast cancer tissue (middle panel) and the normal breast tissue (left panel). In particular, we found in the normal breast tissue and to a lesser extent in the primary breast cancer tissue that mammary epithelial cells displayed an intense and widespread staining for PEDF. All of the normal breast tissue stained positive for PEDF, whereas 68% of primary tumors were PEDF-positive and 32.2% were PEDF-negative. In contrast, we found that 47.6% of recurrence tumors were PEDF-positive and 52.4% (31 out of 59) of recurrence tumors were PEDF-negative (Table 1). The number of recurrence tumors that were PEDF-negative was statistically significantly different from the number of primary tumors that were PEDF-negative (*P *< 0.000001) (Table 1). We also examined PEDF expression in endocrine-responsive tumors (*n *= 150) to assess whether PEDF expression correlated with response to endocrine therapy. We found that ~83.3% of endocrine-responsive tumors were PEDF-positive and 16.7% were PEDF-negative, which was significantly different from the number of recurrence tumors that were PEDF-negative (*P *< 0.000001) or PEDF-positive (*P *< 0.00008) (Table 1). Overall, these data show that patients who had the worst response to endocrine therapy (defined as progressive disease) had significantly lower PEDF expression than those who had the best response to endocrine therapy (defined as complete response) and that poor clinical response to endocrine therapy is associated with PEDF deficiency in primary breast carcinomas. Notably, Cai and colleagues previously reported that PEDF expression was significantly reduced in breast cancer tissues compared with normal breast tissue [24]; however, these investigators did not examine whether PEDF expression correlated with response to endocrine therapy or acquired resistance.

**Figure 2:** **Pigment epithelium-derived factor expression in primary and recurrence breast tumor tissues**. **(a) **Immunohistochemistry (IHC) staining for pigment epithelium-derived factor (PEDF) and estrogen receptor alpha (ERα) were performed on tissue microarrays generated from normal breast tissue (left panel), primary breast tumor tissue (*n *= 59; middle panel), and recurrence breast tumor tissue (*n *= 59; right panel). Cores used to generate tissue microarrays (TMAs) were 0.6 mm in diameter. Tumor tissues were also stained in the absence of a PEDF antibody to act as a negative control (left panel, inset). PEDF staining was quantified as an intensity score ranging from 0 to 255. A scale of 0 to 3 was used to score staining intensity of ERα. **(b) **Western blot analysis of normal tissue (N), primary breast tumor tissue (PT), or recurrence tumor tissue (RT) to assess PEDF, total ERα, and phosphorylated ERα (Ser118 and Ser167) protein level. β-actin was used as a loading control. **(c) **Representative quantitative real-time PCR analysis of *PEDF *and *ER*α mRNA expression in N, PT, or RT. For experiment, total RNA was extracted from paraffin-embedded tissues using Trizol and analyzed by real-time PCR as described in Materials and methods. *PEDF *and *ER*α mRNA were normalized to the internal control gene *PUM1*. All experiments were performed in triplicate. PEDF mRNA level was statistically significantly lower in the recurrence tumor tissue compared with the primary tumor tissue. *P < 0.001.

**Table 1:** Pigment epithelium-derived factor expression in normal versus breast tumor tissue samples

Tissue sample	*n*	PEDF status	Intensity score
Recurrence tumors	28 (47.6%)^a^	Positive	> 150
	31 (52.4%)^b^	Negative	≤ 25
Primary tumors	40 (67.8%)^a^	Positive	> 150
	19 (32.2%)^b^	Negative	≤ 25
Endocrine-responsive tumors	125 (83.3%)^c^	Positive	> 150
	25 (16.7%)^d^	Negative	≤ 25
Normal tissue	5 (100%)	Positive	≥ 200
	0 (0%)	Negative	≤ 25

A total of 209 breast cancer patients were initially treated with tamoxifen and 59 patients developed recurrence disease after a mean follow-up of 93 months. Immunohistochemistry (IHC) staining was performed on tissue microarrays (TMAs) constructed from recurrence breast tumors (*n *= 59) and matched primary breast tumors (*n *= 59). Normal background breast tissue was also used for comparison. TMAs were also constructed from endocrine-responsive tumor tissues (*n *= 150). A semi-automated quantitative image analysis system (ACIS II) was used to quantitate the staining of the TMA slides. For IHC analysis, pigment epithelium-derived factor (PEDF) staining was quantified as an intensity score (scale 0 to 255). ^a^*P *< 0.00003, number of PEDF-positive recurrence tumors versus PEDF-positive primary tumors. ^b^*P *< 0.000001, number of PEDF-negative recurrence tumors versus PEDF-negative primary tumors. ^c^*P *< 0.00008, number of PEDF-positive recurrence tumors versus PEDF-positive endocrine-responsive tumors. ^d^*P *< 0.000001, number of PEDF-negative recurrence tumors versus PEDF-negative endocrine-responsive tumors.

Since loss of ERα has been shown to be associated with the development of endocrine resistance in breast cancer, we assessed ERα status in the primary tumors versus the recurrence tumors using immunohistochemistry. We found that ERα protein was expressed at high levels (+3) in both the primary and the recurrence tumors and that there was no significant difference in ERα expression between the primary versus the recurrence tumors (Figure 2a). Western blot and real-time PCR analyses were also performed on the primary and recurrence breast tumor tissues to determine PEDF and ERα protein and the mRNA status. Figure 2b shows that the PEDF protein level was markedly reduced in the recurrence tumors compared with the primary tumors; however, the total ERα protein level was similar between the two groups with a similar trend observed for PEDF mRNA and ERα mRNA (Figure 2c). We should note that while the total ERα expression level was similar in the primary tumors versus the recurrence tumors, p^ser167^ER protein was markedly elevated in the recurrence tumors versus the primary tumors.

### PEDF silencing confers resistance to tamoxifen in breast cancer cells and its stable expression sensitizes resistant cells to endocrine therapy

To establish a causal connection between PEDF expression and endocrine resistance, we explored the functional consequences of PEDF silencing on tamoxifen sensitivity in endocrine-sensitive MCF-7 and T47D breast cancer cells. Cells were transiently transfected with either PEDF siRNA or nontarget control siRNA for 72 hours and PEDF silencing was quantified by western blot and quantitative RT-PCR analyses. As shown in Figure 3a (top panel), PEDF siRNA dramatically reduced PEDF protein and mRNA levels in both MCF-7 and T47D cells compared with the nontarget control siRNA. PEDF knockdown cells were then treated with 1 μM 4OHT, the active metabolite of tamoxifen, and cell growth was determined after 72 hours using a DNA proliferation assay kit. As shown in Figure 3a (middle panel), PEDF silencing significantly (*P *< 0.01) reduced the sensitivity of MCF-7 and T47D cells to 4OHT compared with cells transfected with the nontarget control siRNA. Specifically, we found that 1 μM 4OHT inhibited the growth of MCF-7 and T47D cells transfected with the nontarget control siRNA by 92% and 87%, respectively, whereas 4OHT reduced the growth in PEDF-knockdown MCF-7 and T47D cells by 45.6% and 54%, respectively. PEDF-knockdown MCF-7 and T47D cells were also treated with 1 μM 4OHT for 72 hours and cell proliferation was determined by counting viable cells using trypan blue exclusion. Figure 3a (bottom panel) showed that 4OHT reduced the proliferation of MCF-7 and T47D cells transfected with the control siRNA by ~85 to 90%; however, in the PEDF knockdown cells, the ability of 4OHT to inhibit proliferation was significantly reduced compared with 4OHT-treated cells transfected with the control siRNA (*P *< 0.01).

**Figure 3:** **Knockdown of pigment epithelium-derived factor expression by siRNA reduces tamoxifen sensitivity in breast cancer cells**. **(a) **siRNA-mediated reduction of pigment epithelium-derived factor (PEDF) expression in MCF-7 and T47D breast cancer cells was performed as described in Materials and methods. Cells were transfected with PEDF or control siRNA for 72 hours and PEDF protein and mRNA levels were determined by western blot and real-time PCR analyses. Transfected cells were also treated with 1 μM 4-hydroxytamoxifen (4OHT) for 72 hours and cell proliferation was determined by DNA quantitation assay and by cell counting using trypan blue exclusion. All experimental points are given as the average of triplicates. **(b) **Stable expression of PEDF in endocrine-resistant MCF-7:5C and BT474 breast cancer cells sensitized them to tamoxifen. A lentiviral construct encoding the human PEDF cDNA was used to stably express PEDF in MCF-7:5C and BT474 cells. Western blot analysis was used to confirm stable expression of PEDF protein in MCF-7:5C and BT474 cells (top panel). To determine the effect of PEDF expression on tamoxifen sensitivity, lentiviral transduced 5C-PEDF and BT474-PEDF cells were treated with 10^-12 ^M to 10^-6 ^M 4OHT for 72 hours and cell proliferation was determined by DNA quantitation assay (middle panel) and by cell counting using trypan blue exclusion (bottom panel). All experimental points are given as the average of triplicates. Assays were performed twice.

Since MCF-7:5C and BT474 breast cancer cells are resistant to tamoxifen and they express low levels of PEDF, we next examined whether stable expression of PEDF in these cells would sensitize them to the inhibitory effects of tamoxifen. We used a lentiviral construct encoding the full-length human PEDF cDNA to stably express PEDF in MCF-7:5C and BT474 cells. The efficiency of PEDF lentiviral transduction of MCF-7:5C and BT474 cells was confirmed by western blot analysis. As shown in Figure 3b (top panel), PEDF expression was very high in the lentiviral transduced cells, 5C-PEDF and BT474-PEDF, compared with the untransduced cells, MCF-7:5C and BT474. Following confirmation of PEDF overexpression, transduced 5C-PEDF and BT474-PEDF cells were treated with 10^-12 ^to 10^-6 ^M of 4OHT for 7 days and cell growth was determined using a DNA quantitation assay. As shown in Figure 3b (middle panel), 4OHT treatment reduced the growth of transduced 5C-PEDF and BT474-PEDF cells in a dose-dependent manner with maximum inhibition at 100 nM compared with untransduced MCF-7:5C and BT474 cells that showed no response to 4OHT at any of the concentrations tested. We confirmed that the inhibitory effect of 4OHT in 5C-PEDF and BT474-PEDF cells was due to a reduction in cell proliferation/viability as determined by trypan blue exclusion and that the re-expression of PEDF in MCF-7:5C and BT474 cells significantly (*P *< 0.05) enhanced their sensitivity to 4OHT compared with the untransduced cells (Figure 3b, bottom panel).

### Effect of PEDF expression on ERα signaling in endocrine-resistant MCF-7:5C cells

Since our tissue microarray data showed increased expression of p^Ser167^ERα in endocrine-resistant tumors that expressed low levels of PEDF, we examined the effect of PEDF re-expression on ERα signaling in endocrine-resistant MCF-7:5C cells that are PEDF-negative. We found that stable expression of PEDF in MCF-7:5C cells (5C-PEDF) dramatically reduced the protein levels of ERα, p^Ser167^ERα, pAKT, and the proto-oncogenic receptor tyrosine kinase RET, which were constitutively elevated in the untransduced MCF-7:5C cells but not parental MCF-7 cells (Figure 4a). Furthermore, we found that treatment of MCF-7:5C cells with 100 nM rPEDF markedly reduced the phosphorylation level of ERα and RET protein in these cells (Figure 4b) and it significantly reduced ERα transcriptional activity in these cells (Figure 4c). In particular, we found that basal ERE luciferase activity was significantly higher (~3.3-fold) in endocrine-resistant MCF-7:5C cells compared with endocrine-sensitive MCF-7 cells and treatment with rPEDF completely suppressed the basal ERE activity in MCF-7:5C cells and it significantly reduced E2-induced ERE activity in these cells (Figure 4c). Noteworthy is that pAKT and RET are known to enhance phosphorylation of ERα at Ser118 and Ser167, which is associated with increased ERα transcriptional activity and tamoxifen resistance [36]. The fact that stable expression of PEDF and the administration of rPEDF protein in MCF-7:5C cells was able to suppress p^Ser167^ERα, p-AKT, and RET expression suggests a potential crosstalk between PEDF, ERα and RET in these cells. This finding highlights a potential mechanism by which silencing/loss of PEDF might contribute to the development of resistance in MCF-7:5C cells. We should note that re-expression of PEDF in BT474 cells did not significantly alter ERα phosphorylation status or RET expression in these cells; however, it did slightly reduce HER2 expression in these cells (data not shown).

**Figure 4:** **Effect of recombinant pigment epithelium-derived factor on the estrogen receptor alpha signaling pathway**. **(a) **Western blot analysis of pigment epithelium-derived factor (PEDF), estrogen receptor alpha (ERα), phospho-ER, phospho-Akt, mitogen-activated protein kinase (MAPK), phospho-MAPK, rearranged during transfection (RET), pRET, p70S6K, and mammalian target of rapamycin (mTOR) protein expression in MCF-7, MCF-7:5C, and 5C-PEDF cells. **(b) **Effect of recombinant PEDF on ERα, pERα, RET, and pRET (Y1062) protein expression in MCF-7:5C cells. Cells were treated with 100 nM recombinant PEDF (rPEDF) protein for 24 hours and cell lysates were analyzed by western blot. β-actin was used as a loading control. **(c) **Effect of rPEDF on estrogen response element (ERE) luciferase activity in MCF-7 and MCF-7:5C cells. MCF-7 and MCF-7:5C cells were grown in estrogen-free RPMI media and then co-transfected with a 5× ERE luciferase plasmid and a renilla reporter plasmid for 24 hours. Following transfection, cells were treated with 1 nM 17β-estradiol (E2), 100 nM rPEDF, or E2 + rPEDF for 24 hours and luciferase activity was measured. Values presented as relative luciferase activity after normalization to *Renilla *luciferase activity. Data expressed as mean ± standard deviation of the results obtained from triplicate experiments. Basal ERE activity was statistically significantly higher in MCF-7:5C cells compared with MCF-7 cells. *P < 0.01.

### Downregulation of RET reverses tamoxifen resistance in MCF-7:5C breast cancer cells

Previous studies have shown that a subset of ERα-positive breast cancers express high levels of mRNA transcripts encoding *RET *and that RET signaling in ERα-positive breast cancer cell lines can result in the activation of MAPK and AKT, which are important regulators of ERα phosphorylation [43,44]. More recently, RET signaling has been implicated in estrogen-independent growth and tamoxifen resistance in breast cancer, potentially through ERα phosphorylation and ligand-independent transcriptional regulation [43-45]. Since our data showed that re-expression of PEDF suppressed RET, ERα and AKT in endocrine-resistant MCF-7:5C cells, we examined the biological effect of RET in endocrine-sensitive MCF-7 breast cancer cells and estrogen-independent and tamoxifen-resistant MCF-7:5C cells. As shown in Figure 5a, RET protein and mRNA levels were markedly increased in endocrine-resistant MCF-7:5C cells compared with MCF-7 cells. Transfection of MCF-7:5C cells with RET siRNA completely downregulated RET protein and mRNA levels (Figure 5b) in these cells. Dose-response survival curves performed over a range of 4OHT concentrations from 10^-9 ^to 10^-6 ^M confirmed that the untreated and siRNA control-treated MCF-7:5C cells were indeed resistant to 4OHT treatment (Figure 5c). In contrast, RET downregulation resulted in a profound increase in sensitivity to 4OHT (Figure 5c). These results indicate that there might be potential crosstalk between PEDF, RET, and ERα signaling pathways and that RET targeting might be a viable strategy to resensitize resistant breast cancers to endocrine therapy.

**Figure 5:** **Knockdown of RET mRNA expression sensitizes endocrine-resistant MCF-7:5C breast cancer cells to 4-hydroxytamoxifen**. **(a) **Rearranged during transfection (RET) protein and mRNA levels in wild-type MCF-7 cells and endocrine-resistant MCF-7:5C cells as determined by western blot analysis and quantitative real-time PCR, respectively. **(b) **MCF-7:5C cells were transfected with either a RET-targeted siRNA or a nontarget control siRNA for 48 hours and *RET *protein and mRNA expression levels were determined by western blotting and real-time PCR. **(c) **Effect of RET suppression on the proliferation of MCF-7:5C cells. Cells were transfected with a RET-targeted or a nontargeting control siRNA, and after 24 hours cells were seeded into 12-well plates and exposed continuously to the indicated concentrations of 4-hydroxytamoxifen (4OHT) or vehicle for an additional 72 hours. Cell proliferation was determined by cell counting using a hemacytometer. Data shown are representative of three independent experiments. UT, untreated.

### PEDF inhibits endocrine-resistant breast cancer cell growth *in vitro *and exhibits anti-tumor activity *in vivo*

Although our studies have shown that PEDF is capable of modulating ERα and RET signaling pathways in endocrine-resistant breast cancer cells, it is worth noting that the most well-known function of PEDF is its ability to inhibit angiogenesis. We therefore examined the effect of rPEDF on the proliferation of endocrine-sensitive MCF-7 and endocrine-resistant MCF-7:5C breast cancer cells. As shown in Figure 6a, rPEDF significantly (*P *< 0.001) reduced the growth of resistant MCF-7:5C cells but had no effect on parental MCF-7 cells. The growth-inhibitory effect of rPEDF was concentration dependent, with maximum inhibition (~90%) observed at 100 nM, and this inhibitory effect of rPEDF was completely blocked by the addition of antibodies specific to PEDF, thus confirming that the effect of PEDF was specific. To determine whether the anti-proliferative effect of rPEDF on MCF-7:5C cells was due to apoptosis, we next performed a TUNEL assay. Figure 6b showed that rPEDF (100 nM) markedly increased apoptosis in MCF-7:5C cells, with 41.8% of cells being TUNEL-positive, compared with the untreated (control) cells that showed very few TUNEL-positive cells. Because rPEDF treatment caused endocrine-resistant MCF-7:5C cells to undergo apoptosis, we also examined whether knockdown of PEDF expression in MCF-7 cells would cause them to undergo apoptosis. We found that PEDF knockdown in MCF-7 cells did not inhibit the growth of these cells or cause them to undergo apoptosis in the presence of rPEDF (data not shown), thus confirming that the ability of rPEDF to induce apoptosis is specific for MCF-7:5C cells.

**Figure 6:** **Effect of recombinant pigment epithelium-derived factor (rPEDF) on the growth of endocrine-sensitive MCF-7 and endocrine-resistant MCF-7:5C breast cancer cells *in vitro *and *in vivo***. **(a) **MCF-7 and MCF-7:5C cells were treated with increasing concentrations of rPEDF, rPEDF + anti-PEDF antibody (anti-PEDF), or anti-PEDF antibody for 7 days, and cell proliferation was determined using a DNA quantitation kit as described in Materials and methods. Experiments were repeated three times, and data are shown as mean ± standard deviation (SD). *P < 0.001 compared with untreated controls. **(b) **MCF-7:5C cells were treated with rPEDF, anti-rPEDF, or rPEDF + anti-rPEDF for 72 hours and apoptosis was determined by TUNEL staining. Bar graph: summary of percentage of apoptotic cells counted in five fields from three experiments. Data presented as mean ± SD. **(c) **Effect of rPEDF on the growth of MCF-7:5C cells *in vivo*. MCF-7:5C cells were bilaterally injected into the mammary fat pad of ovariectomized nude mice, and when tumors reached an area of 0.1 cm^2 ^the mice (*n *= 15/group) were randomized into two treatment groups: PBS or rPEDF. The mean cross-sectional tumor area was measured up to 30 days. Bar graph: mean cross-sectional tumor area in the control group and the PEDF-treated group. **(d) **Intratumoral microvessel density (MVD) in tumor tissues was determined by immunohistochemical staining by an endothelial-specific antibody CD34; PBS group (×200) and PEDF group (×200). Quantitative analysis of microvessel density is also shown. Data presented as mean ± SD.

Since rPEDF was shown to effectively inhibit the growth of endocrine-resistant MCF-7:5C breast cancer cells *in vitro*, we next evaluated the effect of rPEDF on MCF-7:5C tumor growth *in vivo*. Endocrine-resistant MCF-7:5C breast cancer cells were injected subcutaneously into the mammary fat pads of ovariectomized nude mice. When palpable tumors were established (0.1 cm^2^), the animals were randomized into two groups and then treated with either rPEDF (4 mg/kg) or PBS vehicle control that was administered every 2 days by intraperitoneal injection. We found that rPEDF reduced the growth of MCF-7:5C tumors at all of the time points examined. The average tumor area was reduced from 0.42 cm^2 ^in the PBS-treated group to 0.12 cm^2 ^in the rPEDF-treated group (Figure 6c). The differences between the two groups were statistically significant (*P *< 0.001), as calculated by repeated-measures analysis of variance. We next determined whether the anti-tumor activity of rPEDF *in vivo *was due, in part, to its ability to inhibit angiogenesis. For this purpose, MCF-7:5C xenografts were excised at the end of the experiment (day 30) and were sectioned and analyzed by immunohistochemistry using antibody to CD34, a well-known marker for newly formed blood vessels/angiogenesis. As shown in Figure 6d (top), tumors from mice treated with PBS showed intense staining for CD34, indicating the presence of extensive angiogenesis in the tumors, whereas microvessel density in tumors from mice treated with rPEDF was markedly lower. A 48% reduction in microvessel density was observed in the rPEDF-treated group compared with the PBS-treated group (*P *< 0.01; Figure 6d, bottom panel). These data demonstrate that rPEDF is capable of inhibiting the neovascularization of endocrine-resistant breast carcinoma *in vivo*.

### PEDF expression sensitizes endocrine-resistant MCF-7:5C tumors to tamoxifen

Since our *in vitro *data showed that stable expression of PEDF in endocrine-resistant MCF-7:5C cells sensitized them to tamoxifen, we examined whether rPEDF is capable of sensitizing endocrine-resistant MCF-7:5C tumors to tamoxifen in athymic mice. Figure 7a shows that the growth of MCF-7:5C tumors was significantly reduced by rPEDF alone (*P *< 0.0001) but not by tamoxifen alone; however, when rPEDF and tamoxifen were combined the growth of MCF-7:5C tumors was significantly reduced compared with rPEDF alone (*P *< 0.01) (Figure 7a). For comparison, we also performed similar experiments using MCF-7 and BT474 tumors. We found that MCF-7 tumor growth was significantly inhibited by tamoxifen (*P *< 0.0001) and rPEDF (*P *< 0.01); however, the combination of tamoxifen and rPEDF did not further reduce the growth of these tumors compared with the individual treatments (Figure 7b). BT474 tumor growth was also significantly inhibited by rPEDF alone (*P *< 0.001) and the combination of rPEDF and tamoxifen (*P *< 0.05), but tamoxifen alone had no effect (Figure 7c). We next investigated whether ERα and other signaling proteins were altered in MCF-7:5C tumors treated with rPEDF, tamoxifen, or rPEDF and tamoxifen. Western blot analysis of MCF-7:5C tumor extracts showed that p^Ser167^ERα, p-Akt, and p-RET protein were markedly reduced in the rPEDF-treated and rPEDF plus tamoxifen-treated samples compared with control or tamoxifen-treated samples (Figure 7d), which is consistent with our *in vitro *data. Overall, these results suggest that rPEDF is capable of inhibiting the growth of endocrine-sensitive MCF-7 tumors as well as endocrine-resistant MCF-7:5C and BT474 tumors, possibly through its anti-angiogenic activity; however, rPEDF is also capable of sensitizing MCF-7:5C tumors to tamoxifen, which appears to be associated with its ability to downregulate phosphorylated ERα, Akt, and RET in these tumors.

**Figure 7:** **Effect of recombinant pigment epithelium-derived factor on tamoxifen sensitivity in MCF-7:5C, MCF-7, and BT474 xenografts**. **(a) **MCF-7:5C cells were bilaterally injected into the mammary fat pads of ovariectomized athymic mice (*n *= 32), and after tumors reached a mean cross-sectional area of 0.2 cm^2 ^groups of eight mice were randomly assigned to the following treatments: PBS (control), recombinant pigment epithelium-derived factor (rPEDF), tamoxifen (TAM), or rPEDF + TAM. TAM was given orally by gavage at 1.5 mg/day and rPEDF was given via intraperitoneal injection at 4 mg/kg every other day for 21 days. **(b) **MCF-7 cells were bilaterally injected into the mammary fat pads of ovariectomized mice (*n *= 32), and after tumors reached a mean cross-sectional area of 0.32 cm^2 ^groups of eight mice were randomly assigned to the following treatments: PBS (control), rPEDF, TAM, or rPEDF + TAM as described in Materials and methods. **(c) **BT474 cells were bilaterally injected into the mammary fat pads of ovariectomized mice (*n *= 32), and after tumors reached a mean cross-sectional area of 0.3 cm^2 ^groups of eight mice were randomly assigned to the following treatments: PBS (control), rPEDF, TAM, or rPEDF + TAM. Mean cross-sectional tumor area was measured every 5 days with vernier calipers. Cross-sectional areas were calculated by multiplying the length (*l*) by the width (*w*) and by π and dividing the product by 4 (that is, *lw*π/4). **(d) **Western blot analysis of MCF-7:5C tumors following treatment with rPEDF, tamoxifen, or rPEDF and tamoxifen. Tumors were generated as described in 7a and the lysates were preprepared as described in Materials and Methods. Blots were probed with the indicated antibodies.

## Discussion

Resistance to endocrine therapy presents a major challenge in the management of ERα-positive breast cancer and is an area under intense investigation. While many studies point towards the cross-talk between ERα and growth factor receptor signaling pathways as the key in the development of resistance [5,6,46,47], the underlying mechanism is still not fully understood and, as a consequence, effective approaches for preventing and overcoming resistance are not yet available. PEDF is a secreted glycoprotein that was first described in the late 1980s after it was identified and isolated from conditioned medium of cultured primary human fetal retinal pigment epithelial cells [8]. PEDF is ubiquitously expressed in many tissues and possesses potent anti-angiogenic activity, being more than twice as potent as angiostatin and more than seven times as potent as endostatin [12]. Recent studies indicate that PEDF expression is significantly reduced in a wide range of tumor types and that its re-expression in these tumors delays the onset of primary tumors and decreases metastases [48]. In the present study, we show that loss of PEDF expression in breast cancer is associated with the development of endocrine resistance and that there is functional crosstalk between PEDF and the ERα signaling pathway. Specifically, we found that PEDF protein and mRNA levels were markedly reduced in tamoxifen-resistant breast tumors and in breast cancer cells that are resistant to AIs and/or tamoxifen. We also found that stable re-expression of PEDF in the resistant cells re-sensitized them to the antiproliferative effects of tamoxifen and that re-expression of PEDF dramatically reduced the expression of the receptor tyrosine kinase RET along with p-AKT and p^Ser167^ERα. Furthermore, we found that exogenous administration of rPEDF significantly inhibited the growth of endocrine-resistant breast cancer cells *in vitro *and *in vivo *but had no effect on the growth of endocrine-sensitive breast cancer cells *in vitro *with marginal effect *in vivo*. While PEDF is known to exert anti-tumor activity by inhibiting angiogenesis [49,50] and inducing apoptosis [17], the present study is the first to demonstrate a link between loss of PEDF expression and the development of endocrine resistance and to show that PEDF re-expression is capable of reversing tamoxifen resistance in breast cancer.

During the past decade, researchers have prepared various forms of PEDF and demonstrated its beneficial effects in several tumor models. Doll and colleagues reported that exogenous rPEDF protein induced tumor epithelial apoptosis in mouse prostate and pancreas [13]. Liu and colleagues showed that a short peptide derived from the parent PEDF molecule was able to inhibit osteosarcoma growth [51]. Hase and colleagues demonstrated that intratumoral injection of a lentivirus vector encoding PEDF resulted in inhibition of human pancreatic cancer in nude mice [52]. Moreover, Wang and colleagues showed that *in vivo *transfer of PEDF mediated by adenoviral vectors exerted a dramatic inhibition of tumor growth in athymic nude mice implanted with the human HCC and in C57BL/6 mice implanted with mouse lung carcinoma [53]. In the present study we showed that exogenous rPEDF preferentially induced apoptosis in endocrine-resistant MCF-7:5C and BT474 breast cancer cells compared with endocrine-sensitive MCF-7 cells and that rPEDF partially reversed the tamoxifen-resistant phenotype of MCF-7:5C and BT474 cells *in vitro *and *in vivo*. Interestingly, we found that lentiviral-mediated re-expression of PEDF in the resistant cells also reversed tamoxifen resistance in these cells. Investigation into the mechanism of action of PEDF in the resistant cells indicated that the anti-tumor activity of PEDF in *vivo *was due, in part, to its ability to inhibit angiogenesis, as was demonstrated by a reduction in microvessel density and an increase in apoptosis. Interestingly, we found that exogenous PEDF failed to induce apoptosis in MCF-7 breast cancer cells *in vitro*; however, it significantly inhibited the growth of MCF-7 tumors in athymic mice, which was due to its anti-angiogenic activity. The anti-tumor activity of PEDF, however, was more pronounced in the endocrine-resistant breast cancer cells compared with the endocrine-sensitive cells. We should note that a similar finding was reported by Konson and coworkers in which they showed that exogenous PEDF preferentially induced apoptosis in endothelial cells compared with MDA-MB-231, HCT116, and U87-MG cancer cells [54,55]; however, PEDF efficiently inhibited the growth rate of xenografts generated from these cancer cells. While the reason for this cell-type specific effect of PEDF is not known, there is evidence for multiple PEDF receptors at the cell surface including the recently identified non-integrin 67/37-kDa laminin receptor [56], extracellular matrix components [57], and a phospholipase-linked membrane protein [58]. Differential expression of these receptors on neuronal, endothelial, and cancer cells may provide a partial explanation for the differential effects on these cell populations. Identification of which of these PEDF receptors are present on cancer cells, as well as further elucidation of signaling downstream of PEDF, could lead to the identification of new pharmacologic targets for both anti-cancer and neuronal survival therapies. We are currently trying to determine whether there is a specific PEDF receptor expressed in breast cancer cells and whether the functional activity of the receptor is altered by the endocrine responsiveness of the cells.

Apart from its ability to inhibit to angiogenesis, we also found that PEDF suppressed RET expression in endocrine-resistant breast cancer cells and that this suppression was associated with the reversal of tamoxifen resistance. Specifically, we found that basal RET, p-RET, ERα, and p^Ser167^-ERα protein levels were markedly increased in endocrine-resistant MCF-7:5C cells compared with endocrine-sensitive MCF-7 cells and stable expression of PEDF in MCF-7:5C cells or treatment of these cells with rPEDF-suppressed RET, p-RET, and p^Ser167^-ERα protein in these cells. Furthermore, we found that suppression of RET expression using siRNA knockdown also reversed tamoxifen resistance in MCF-7:5C cells, which suggests a role for RET in tamoxifen resistance. This finding is important because recent studies have indicated that RET is involved in the biology of ERα-positive breast cancers [43,44] and in the response to endocrine treatment [45]. Two independent studies have identified RET overexpression in a subset of ERα-positive breast cancers [43,44], suggesting an important role of RET in this subset. By *in situ *hybridization, in a cohort of 245 invasive breast cancers, RET mRNA was detected in 29.7% of the tumors and preferentially expressed in ER-positive cases. Subsequent studies in the same cohort of patient samples corroborated that increased RET mRNA levels correlated with increased RET protein expression. Similar findings were reported for many breast cancer cell lines where RET expression correlated strongly with ERα expression and/or ErbB2/HER2 overexpression [43].

RET is a receptor tyrosine kinase protein of 150 kDa that is expressed and required during early development for the formation of neural crest-derived lineages, kidney organogenesis, and spermatogenesis [59]. RET is considered the driving oncogene in various neoplasms of the thyroid, where specific mutations lead to defined tumor types [60-62]. The RET protein spans the cell membrane, so that one end of the protein remains inside the cell and the other end projects from the outer surface of the cell. This positioning of the protein allows it to interact with specific factors outside the cell and to receive signals that help the cell respond to its environment. When molecules that stimulate growth and development such as growth factors attach to the RET protein, a complex cascade of chemical reactions inside the cell is triggered. These reactions instruct the cell to undergo certain changes, such as dividing or maturing to take on specialized functions. RET is the receptor for a family of glial-derived neurotrophic factor (GDNF) ligands, which includes GDNF, artemin, neurturin, and persephin [60,63]. These ligands bind RET in conjunction with glycosylphosphatidylinositol-anchored co-receptors of the GDNF receptor alpha family, and the ligand-co-receptor-RET complex formation results in transient RET dimerization and activation of the RET tyrosine kinase domain. RET protein dimerization results in autophosphorylation of several intracellular RET tyrosine residues, and these autophosphorylation sites serve as binding sites for a variety of docking proteins. In particular, the tyrosine Y1062 has been shown to bind Src homology and collagen, insulin receptor substrate1/2, fibroblast growth factor receptor substrate 2, and protein kinase C alpha. These proteins are able to activate multiple signaling pathways, including MAPK, PI3K/AKT, RAS/extracellular signal-regulated kinase and Rac/c-*jun *NH kinase, which are mediators of cell motility, proliferation, differentiation, and survival [64]. While our present study indicates that PEDF is capable of suppressing RET signaling in endocrine-resistant cells, we do not know the exact mechanism by which this occurs. We should note that RET is the receptor for several ligands including GNDF, which is a potent neurotropic factor similar to PEDF. Like other trophic factors, PEDF is thought to exert its biological effects by specifically binding and activating one or more receptors. While PEDF receptors have not yet been fully characterized, there is a possibility that PEDF, like GDNF, is able to bind to RET and thus regulate its expression and activity in breast cancer cells. This possibility is currently being investigated in our laboratory.

RET and other growth factor receptor tyrosine kinases are known to activate ERα through phosphorylation [36]. The ERα contains two distinct transcription activation domains, AF-1 and AF-2, which can function independently or synergistically. AF-2 is located in the ligand-binding domain region of ERα and its activity is dependent on estrogen binding, whereas AF-1 activity is regulated by phosphorylation that can occur independently of estrogen binding [5]. The extracellular signal-regulated kinase 1/2 pathway phosphorylates ERα directly and/or via p90RSK, whereas AKT phosphorylates ERα directly and/or via mTOR. In contrast, RET increases ERα phosphorylation at Ser118 and Ser167 through activation of the mTOR/p70S6K pathway [43,59,65], which can be independent of the PI3K/AKT pathway. Notably, p70S6K, mTOR, and p-AKT were also constitutively overexpressed in endocrine-resistant MCF-7:5C cells prior to stable expression of PEDF in these cells. In addition, basal ERα transcriptional activity, as determined by ERE luciferase assay, was significantly elevated in MCF-7:5C cells compared with wild-type MCF-7 cells, and treatment of these cells with rPEDF inhibited phosphorylation of ERα and RET and suppressed the basal ERE activity in these cells. Interestingly, we found that suppression of RET expression using siRNA and inhibition of the mTOR pathway using rapamycin was able to reverse tamoxifen resistance in MCF-7:5C cells; however, inhibition of the PI3K/AKT pathway in these cells did not reverse their tamoxifen-resistant phenotype but it did reduce their hormone-independent growth. Notably, crosstalk between RET and ERα has previously been reported by Plaza-Menacho and coworkers, who showed that activation of RET by its ligand GDNF increased ERα phosphorylation on Ser118 and Ser167 and increased estrogen-independent activation of ERα transcriptional activity [45]. Further, they identified mTOR as a key component in this downstream signaling pathway and they showed in tamoxifen-resistant (TAM_R-_1) MCF-7 cells that targeting RET restored tamoxifen sensitivity.

## Conclusion

In summary, we have found that PEDF expression is markedly reduced in endocrine-resistant breast cancer and that stable expression of PEDF in endocrine-resistant cells restores their sensitivity to tamoxifen by suppressing RET and ERα signaling. The ability of PEDF to suppress RET signaling in endocrine-resistant cells is a newly identified function of PEDF that is independent of its most well-known function as a potent endogenous anti-angiogenic factor. This finding suggests that PEDF expression in breast cancer might be an important marker of endocrine responsiveness and that loss of PEDF might be a potential hallmark for the development of endocrine resistance. The fact that PEDF is endogenously produced and is widely expressed throughout the body reduces the likelihood that it will have adverse side effects like other synthetic agents or develop drug resistance. However, we should caution that relatively little is known of the overall physiologic role of PEDF in the human body; hence, further investigation is required before any clinical trial can be initiated.

## Abbreviations

AI: aromatase inhibitor; DMEM: Dulbecco modified eagle's medium; ER: estrogen receptor; ERE: estrogen response element; E2: 17β-estradiol; FBS: fetal bovine serum; GDNF: glial cell-derived neurotrophic factor; 4OHT: 4-hydroxytamoxifen; iRNA: interfering RNA; MAPK: mitogen-activated protein kinase; mTOR: mammalian target of rapamycin; PBS: phosphate-buffered saline; PCR: polymerase chain reaction; PEDF: pigment epithelium-derived factor; PI3K: phosphoinositide 3-kinase; rPEDF: recombinant pigment epithelium-derived factor; RET: rearranged during transfection; RT: reverse transcriptase; siRNA: small interfering RNA; TUNEL: terminal deoxynucleotidyl transferase-mediated dUTP nick end-labeling.

## Competing interests

The authors declare that they have no competing interests.

## Authors' contributions

RJ performed the *in vitro *studies. MH constructed the tissue microarrays and performed all of the immunohistochemistry experiments. JL-W conceived the study, participated in the research design and implementation of the study, analyzed and interpreted the data, and drafted the manuscript. All authors read and approved the final manuscript for publication.
